# The Effect of Human Bone Marrow Mesenchymal Stem Cell-Derived Exosomes on Cartilage Repair in Rabbits

**DOI:** 10.1155/2022/5760107

**Published:** 2022-09-08

**Authors:** Hongwei Yang, Meng Cong, Weixiao Huang, Jin Chen, Min Zhang, Xiaosong Gu, Cheng Sun, Huilin Yang

**Affiliations:** ^1^Department of Orthopedics, The First Affiliated Hospital of Soochow University, Suzhou 215006, China; ^2^Orthopedic Institute, Soochow University, Suzhou 215007, China; ^3^Department of Orthopedics, Affiliated Nantong Hospital 3 of Nantong University, Nantong 226001, China; ^4^Key Laboratory of Neuroregeneration of Jiangsu and Ministry of Education and Co-Innovation Center of Neuroregeneration, Nantong University, 19 Qixiu Road, Nantong 226001, China; ^5^Department of Orthopedics, Affiliated Hospital of Nantong University, Nantong 226001, China

## Abstract

Mesenchymal stem cells (MSCs) have shown chondroprotective effects in cartilage repair. However, side effects caused by MSC treatment limit their application in clinic. As a cell-free therapy, MSC-derived exosomes (EXOs) have attracted much more attention in recent years. In the present study, we prepared EXOs from human bone marrow mesenchymal stem cells (hBMSCs) and examined their therapeutic potentials in cartilage repair. Our results showed that the prepared extracellular vesicles exhibit classical features of EXOs, such as cup-like shape, around 100 nm diameter, positive protein markers (CD81, TSG101, and Flotillin 1), and ability of internalization. In primary chondrocytes, the treatment of hBMSC-EXOs markedly increases cell viability and proliferation in a dose-dependent manner. Moreover, wound healing assay showed that hBMSC-EXOs accelerate cell migration in primary chondrocytes. JC-1 staining revealed that the mitochondrial membrane potential was enhanced by hBMSC-EXOs, indicating cell apoptosis was decreased in the presence of hBMSC-EXOs. In rabbits with articular cartilage defects, local administration with hBMSC-EXOs facilitates cartilage regeneration as evidenced by gross view and hematoxylin-eosin (H&E) and Saf-O/Fast Green staining. In addition, the International Cartilage Repair Society (ICRS) score was increased by the application of hBMSC-EXOs. Overall, our data indicate that the treatment with hBMSC-EXOs is a suitable cell-free therapy for treating cartilage defects, and these benefits are likely due to improved cell proliferation and migration in chondrocytes.

## 1. Introduction

Cartilage is a connective tissue with an important role for keeping joints lubricated to ensure smooth movement [1]. Unlike most other tissues, cartilage is composed of gelatinous matrix such as collagen proteins, which were mainly synthesized by chondrocytes. Of note, cartilage has no blood vessels or nerves. Therefore, cartilage regeneration is a tough task due to limited nutrient supply [2]. Cartilage dysfunctions such as defects and injuries often happen that are causative factors for osteoarthritis [3]. Therefore, functional recovery in articular cartilage after injury is a big challenge. Traditional treatments for articular cartilage repair, including nonsteroidal anti-inflammatory drugs, corticoids, acetaminophen, and hyaluronic acid, only ameliorate the symptoms and have marginal effects on cartilage regeneration [4]. Most recently, several strategies were developed for dealing with cartilage defects, including implantation of chondrocytes, osteochondral autograft, and cartilage allograft [5]. However, these mentioned drugs and newly developed strategies still cannot fully resolve cartilage defects in clinic [6]. Hence, alternative strategies aimed at cartilage regeneration are urgently required.

Mesenchymal stem cells (MSCs) have shown promising benefits for cartilage repair due to their potent capacity in differentiation into various types of cells [7]. MSCs could be induced into chondrocyte-like cells to produce extracellular matrix for cartilage regeneration [8]. In addition, MSCs could secrete anti-inflammatory cytokines to modulate immune response, by which a favorable microenvironment was constructed during cartilage repair [9]. To date, MSCs from different sources including bone marrow [10], adipose tissue [11], peripheral blood [12], umbilical cord blood [13], and umbilical cord [14] have been shown promising effects in cartilage tissue engineering. Of them, bone marrow MSCs are considered as the preferred seed cells for treating osteochondral defects due to their advantages in proliferation, chondrogenic differentiation, and easy collection [15]. However, several shortcomings including low survival rate *in vivo* and potential immune rejection impede their application in clinic [16].

Exosomes (EXOs) are small extracellular vesicles with the diameter ranging from 30 to 150 nm, which hold great potentials in translation medicine by delivering functional molecules to treat various disorders [17]. The benefits of MSC-based therapies in tissue repair have been ascribed to the secreted trophic factors, in which EXOs may play a pivotal role. It has been shown that, similar to MSCs, MSC-derived EXOs also have similar effects in tissue repair [18]. Hence, EXOs produced by MSCs, instead of MSCs themselves, were widely used in tissue repair due to the fact that direct use of MSCs may cause side effects such as chromosomal variations and immune rejection [19]. As for cartilage repair, several studies have demonstrated the therapeutic potentials of MSC-derived EXOs. For instance, EXOs from human embryonic MSCs improved cartilage regeneration after injury in rats and micropigs [20, 21]. Articular cartilage repair was enhanced by kartogenin-pretreated infrapatellar fat pad MSC-derived EXOs [22]. EXOs derived from human MSCs promoted cartilage repair and chondrocyte proliferation in osteoarthritis in rats [23]. However, there are several unresolved aspects regarding this newly emerged therapy, including source of MSCs, EXO delivery method and dosage, and the underlying molecular mechanisms.

In this study, therefore, we examined the effects of human bone marrow mesenchymal stem cell- (hBMSC-) derived EXOs on cartilage repair in rabbits. Our results showed that EXOs from hBMSCs greatly improved cartilage repair after injury, and these benefits are likely due to EXOs' induced cell viability, proliferation, and migration in chondrocytes. These data suggest that EXOs derived from hBMSCs hold great therapeutic potentials for treating cartilage dysfunction-associated diseases.

## 2. Materials and Methods

### 2.1. Isolation and Culture of hBMSCs

Human bone marrow samples were obtained from Nantong Third People's Hospital. Bone marrow samples were harvested from the iliac crest of six normal human donors (mean age: 38 years old with the range from 33 to 43). The study was approved by the Institutional Review Board of the Affiliated Nantong Hospital 3 of Nantong University (IRB No. EL2022009). All participants gave written informed consent. The procedures for BMSC isolation were described previously [24]. Briefly, 2 ml human bone marrow was mixed with 8 ml alpha-modified Eagle's medium (*α*-MEM) (HyClone; SH30265.01), in which 10% fetal bovine serum (FBS; Sigma) and 1% penicillin-streptomycin (Beyotime; C0222) were supplemented. The mixture was then added into 100 mm cell culture dish and cultured at 37°C with 5% CO_2_ atmosphere. After 4 days, cell culture medium was refreshed to remove nonadherent cells. The remaining attached cells were considered as hBMSCs. Cells were passaged at 80% confluence by adding 0.25% trypsin. Passage 3-4 (P3-P4) cells were used for experiments [25].

### 2.2. hBMSC-EXO Isolation and Identification

Exosomes (EXOs) were extracted from cell culture supernatant of hBMSCs. For isolating EXOs, culture medium was switched to serum-free medium for 48 h after cells reached 80% confluence. The supernatant was collected and centrifuged at 500*g* for 10 min to remove cell debris, followed by filtration with a 0.22 *μ*m filter (Millipore). EXOs were isolated using an exoEasy Kit (QIAGEN; 76064) from 15 ml cell culture supernatant according to the manufacturer's protocol. Briefly, filtered supernatant was carefully transferred to a new tube. Then, 1 volume of buffer XBP was added to cleared supernatant. After that, a total of 30 ml of mixture was added onto the exoEasy spin column and centrifuged at 500*g* for 1 min. After discarding the flow-through, the column was placed back into the same collection tube. The above steps were repeated until the cleared supernatant was no more than 2 ml. Then, 10 ml of buffer XWP was added to the spin column and centrifuged to remove residual buffer at 5000*g* for 5 min. Transfer the spin column to a fresh collection tube. Add 400 *μ*l buffer XE to the membrane and incubated for 1 min. The eluate was collected by centrifuging at 500*g* for 5 min. Add the eluate to the spin column and incubated for 1 min again. Finally, collect the eluate after centrifugation at 5000*g* for 5 min. Carefully resuspend the resulting EXOs in sterilized PBS and store at -80°C until use.

Morphology of EXOs were observed with a transmission electron microscope (TEM, Hitachi). EXO diameter and particle number were analyzed by nanoparticle tracking analysis (NTA, German Particle Metrix) with the software of Zeta View 8.05.04 (German Particle Metrix). Protein concentration was measured using a bicinchoninic acid (BCA) assay kit (Pierce; 23225). Exosomal markers CD81 (Abcam; ab79599), Flotillin 1 (Abcam; ab133497), and tumor susceptibility gene 101 (TSG101; Abcam; ab125011) were examined by western blot analysis [26].

### 2.3. Rabbit Primary Chondrocyte Culture and Treatment

To isolate primary chondrocytes, 4-week-old New Zealand white rabbits were used. The terminal of tibia and femur was collected for preparing cartilage slices. After 3-time washing in PBS, the slices were incubated with 0.25% trypsin for 0.5 h, and then, 0.2% collagenase II (Sigma-Aldrich; V900892) was added and digestion was performed at 37°C for 12 h. After digestion, the samples were filtered using a strainer (200-mesh). The resulting filtrate was subjected to 5 min centrifugation at 190*g*. The residue containing primary chondrocytes was then resuspended in DMEM/F12 medium containing 10% FBS and plated in flasks. P1 chondrocytes were analyzed by immunofluorescence analysis of collagen II. P2 chondrocytes were used for experiments [27]. To evaluate the potential roles of hBMSC-derived EXOs in chondrocytes, the prepared EXOs at different dosages were added into cell culture medium directly.

### 2.4. Cell Viability Assay

Chondrocytes were seeded in a 96-well plate at 5 × 10^3^ cells/well and cultured in a cell incubator for 6 h. Cells were treated with exosomes at different dosages (2.5 × 10^8^/ml, 5.0 × 10^8^/ml, 1.0 × 10^9^/ml, and 2.0 × 10^9^/ml) for 24 h or 48 h. Cell viability was assayed using a cell counting kit-8 (Dojindo Molecular Technologies; CK04) with the manufacturer's specifications. With a microplate reader (BIOTEK), optical density at 450 nm was measured.

### 2.5. Cell Proliferation Assay

Cell proliferation was analyzed with a 5-ethynyl-20-deoxy uridine (EdU) labeling kit (Ribobio; C10310-3). 50 *μ*M EdU was added to culture medium, and 2 h incubation was performed. After rinsing two times in PBS, cells were then subjected to 30 min fixation in 4% paraformaldehyde. Glycine (2 mg/ml) was added and incubated for 5 min to remove the aldehyde group. After washing in PBS, cells were incubated with the Apollo staining solution. 30 min postincubation, staining solution was removed and cells were treated with 0.5% Triton X-100 for 10 min. Hoechst 3342 was used to stain the nuclei. Cell images were taken with a fluorescence microscope (Life Technology; EVOS FL Auto). Cell proliferation was analyzed by the percentage of EdU-positive cells.

### 2.6. Mitochondrial Membrane Potential Measurement

A JC-1 kit (Beyotime; #C2005) was used to detect mitochondrial membrane potential of chondrocytes. In a 24-well plate, cells were seeded and treated with EXOs (1.0 × 10^9^/ml) at 37°C for 24 h or 48 h. Cells were then subjected to JC-1 staining via incubation in the working solution for 20 min, and then, a fluorescence microscope (Life Technology; EVOS FL Auto) was used to observe and take images of cells. Fluorescence intensity was analyzed by the software of ImageJ.

### 2.7. Scratch Wound Healing Assay

Cell migration was analyzed by wound healing assay [28]. A culture-insert plate (ibidi GmbH) was used in this assay, in which chondrocytes were seeded at 2 × 10^4^ cells per well. 12 h postseeding, the culture insert was removed and nonadherent cells were removed after washing in PBS. Then, cells were incubated with EXOs (1.0 × 10^9^/ml) and photographed at 24 and 48 h post-EXO treatment. With a light microscope, migrated cell numbers were manually counted. For each well, three fields were subjected for counting. The areas were determined using the ImageJ software (National Institutes of Health, USA).

### 2.8. Exosome Internalization Assay

PKH26 (Sigma-Aldrich; PKH26PCL) was used for labeling EXOs according to the manufacturer's instructions. Excess dye was eliminated by centrifugation at 5000*g* for 17 min at 4°C using Amicon Ultra-15 tube (Millipore; UFC9050). After 3-time washing in PBS, the pellets were resuspended in PBS and designated as labeled EXOs. For internalization, EXOs were cocultured with rabbit chondrocytes at 1 × 10^9^/ml in serum-free medium at 37°C. 3, 6, 12, 24, 48, and 72 h postincubation, cells were fixed with 4% paraformaldehyde. The nuclei were stained with DAPI, and the cytoskeleton was stained by FITC-Phalloidin (Sigma-Aldrich; P5282). Internalization of EXOs was monitored with a confocal microscope (Zeiss LSM710, Germany).

### 2.9. Osteochondral Defect Model in Rabbits

Six-month-old male New Zealand white rabbits were provided by the Animal Center of Nantong University. Animals were randomly allocated into four groups: normal group (*n* = 6), PBS group (*n* = 6), low-dosage EXO group (*n* = 6), and high-dosage EXO group (*n* = 6). After anesthetization, rabbits were subjected to surgery to construct cylindrical defects (4 mm × 3 mm; diameter × depth) in the patellar groove of left posterior [29]. To avoid infection, penicillin was given to rabbits at the dosage of 70 mg/kg/day for 3 days via intramuscular injection after the incisions were closed. For pain relief, rabbits received oral meloxicam at the dosage of 0.2 mg/kg/day for 3 days after surgery. One week later, rabbits in the EXO group received 300 *μ*l of 1 × 10^10^ particles/ml (low dosage) or 5 × 10^10^ particles/ml (high dosage) by intra-articular injection. Animals in the PBS group were administered 300 *μ*l of PBS. These treatments were performed once a week and lasted for 4 weeks. At the 5th week, rabbit knee joints were collected for further analysis after sacrifice. All animal protocols were approved by the Ethics Committee of Nantong University and the Jiangsu Province Animal Care Ethics Committee (Approval ID: SYXK [SU] 2017-0046).

### 2.10. Histological Staining and Evaluation of Cartilage Repair

Tissues were fixed in 4% paraformaldehyde for 24 h, and then, tissues were subjected to 30-day decalcification in 10% EDTA (pH 7.4). Tissues were then cut into 5 *μ*m thick sections after embedding in paraffin. With 200 *μ*m intervals, the medial and lateral compartments were used for tissue sectioning. After being deparaffinized in xylene, sections were rehydrated using a graded series of ethanol. Thereafter, Safranin O/Fast Green staining (Solarbio; G1371-5) and hematoxylin and eosin staining (H&E) were performed. Sample collection and photographing were described elsewhere [30]. Cartilage repair was evaluated by the International Cartilage Repair Society (ICRS) scoring standard [31].

### 2.11. Statistical Analysis

The presented data were presented as mean ± SEM from at least three independent experiments. Statistical significance was analyzed using GraphPad Prism software (Version 9.0.0; San Diego, CA, USA). One-way analysis of variance (ANOVA) with Bonferroni's post hoc test was used for statistical analysis. *P* < 0.05 was considered statistically significant.

## 3. Results

### 3.1. Identification of hBMSCs and hBMSC-derived EXOs

In the present study, hBMSCs were prepared from healthy donors and were used for preparing EXOs. Transmission electron microscope (TEM) images showed that EXOs derived from hBMSCs had a cub-like shape coated with bilayer membranes (Figure 1(a)). Nanoparticle tracking analysis (NTA) revealed that the average diameter of prepared EXOs was 131.2 nm, and the EXO concentration was around 1.2 × 10^11^ particles/ml (Figure 1(b)). Furthermore, the positive markers of EXOs such as CD81, TSG101, and Flotillin 1 were expressed in hBMSC-EXOs, while *β*-Actin was only detected in the total cell lysates of hBMSCs (Figure 1(c)). Next, we tested the ability of internalization of these EXOs. To this end, we isolated primary chondrocytes from rabbits, which highly expressed collagen II (Figure 1(d)). As shown in Figure 1(e), EXOs labeled with PKH26 were gathered in rabbit primary chondrocytes according to the confocal microscope images. These data clearly indicate that the prepared extracellular vesicles from hBMSCs are EXOs.

### 3.2. hBMSC-EXOs Facilitate Cell Proliferation in Chondrocytes

Next, we examined the potential roles of hBMSC-EXOs in primary chondrocytes. The results showed that, after 24 h or 48 h incubation, EXOs markedly promoted cell viability in chondrocytes in a dose-dependent manner (Figure 2(a)). EdU incorporation assay showed that cell proliferation was significantly enhanced by high dose of EXOs (1 × 10^9^/ml) at both 24 h and 48 h (Figures 2(b) and 2(c)). These data indicate that hBMSC-EXOs are capable of promoting cell viability and proliferation in primary chondrocytes.

### 3.3. hBMSC-EXOs Enhance Cell Migration and Inhibit Apoptosis in Chondrocytes

Moreover, we also employed wound healing assay to analyze cell migration. The results showed that hBMSC-EXOs accelerated the motility of chondrocytes after 24 h or 48 h incubation (Figures 3(a) and 3(b)). JC-1 is a novel dye for evaluating the mitochondrial membrane potential. A monomer with green fluorescence was presented at low concentrations for this dye. At high concentrations, JC-1 exists as aggregates with an emission maximum at around 590 nm. Our data showed that the treatment of EXOs reduced JC-1 monomers in chondrocyte as evidenced by decreased green fluorescence intensity (Figure 3(c)). Meanwhile, JC-1 aggregates were increased in chondrocytes due to enhanced red fluorescence intensity (Figure 3(c)). As a result, the ratio between red to green fluorescence intensity was improved by hBMSC-EXOs (Figure 3(d)). These data indicate that EXOs derived from hBMSCs have an ability for promoting the cell migration and inhibiting apoptosis in chondrocytes.

### 3.4. hBMSC-EXOs Promote Cartilage Repair after Injury in Rabbits

The above data showed that hBMSC-EXOs hold benefits in chondrocytes, such as increasing cell viability and proliferation and stimulating the mitochondrial function and cell migration. These observed benefits prompt us to examine whether they have similar functions *in vivo*. To select an appropriate regimen in animal experiments, we first examined the time course effect of exosome internalization in chondrocytes. The endocytosis of EXOs by chondrocytes occurred at 3 h, and thereafter, it was gradually increased till 72 h (Figures 4(a) and 4(b)). Since there is severe overlap of growing cells, we did not extend the test time. Based on these findings, we predicted that the endocytosis of hBMSC-EXOs in chondrocytes may peak at 3-4 days postincubation. Therefore, we adopt the regimen in which hBMSC-EXOs were given to the rabbits once a week. To investigate the role of hBMSC-EXOs in cartilage repair in vivo, we generated osteochondral defect model in rabbits; a cylindrical defect with 4 mm × 3 mm (diameter × depth) was created in the patellar groove. Histological analysis was conducted after a 4-week treatment with hBMSC-EXOs. The whole experimental design is illustrated in Figure 5(a). According to the gross view and H&E staining, the defects still could be seen in the PBS group; however, the treatment of hBMSC-EXOs exhibited visible cartilage repair especially in rabbits treated with higher dosage of EXOs (Figures 5(b) and 5(c)). The Saf-O/Fast Green staining further confirmed that the articular cartilage defects in rabbits were largely improved by hBMSC-EXOs (Figure 6(a)). Meanwhile, we also evaluated cartilage regeneration by using the ICRS visual histological score system. Histological assessment was performed in a blinded manner by the same two independent observers. The scores in the EXO group were markedly improved with comparison to those in the PBS group. Of note, the score was further increased by high dosage of hBMSC-EXOs (Figure 6(b)), which was consistent with the histological staining as mentioned above.

## 4. Discussion

Cartilage is a flexible tissue, which is mainly composed of water and several types of proteins including proteoglycans, collagens, and noncollagenous proteins. Of note, these specialist proteins are produced by a group of cartilage cells called chondrocytes. Therefore, chondrocytes are extremely important for proper functioning of cartilage. To evaluate the effects of hBMSC-EXOs in cartilage repair, we first analyzed the effects of hBMSC-EXOs on chondrocytes. Our data showed that the cell proliferation and migration in chondrocytes were promoted by hBMSC-EXOs. Chondrocyte proliferation and migration are two essential events for maintaining healthy cartilage. In line with our findings, other source EXOs also hold capacity for stimulating cell migration and proliferation in chondrocytes [32–35]. Recently, rat BMSC-derived EXOs have shown to protect chondrocytes from advanced glycation end product-induced damages [36]. EXOs from human urine-derived stem cells (hUSCs) are capable of inducing proliferation and migration in chondrocytes [37]. Moreover, human MSCs-EXOs were found to inhibit autophagy and apoptosis in chondrocytes by activating the axis of PI3K/Akt/mTOR [38]. Mitochondria are the power supply center of the cell, providing ATP in many key biological events, such as cell growth, differentiation, and migration [39]. Defects in mitochondrial function and damages induced by oxidative stress are causative factors for loss of chondrocytes in cartilage defects [40]. In the present study, we treated chondrocytes with hBMSC-EXOs and found that this treatment greatly improves mitochondrial activity. One previous study also showed that EXO-derived MSCs inhibit mitochondrial dysfunction and reduce chondrocyte apoptosis [41].

To date, numerous studies examined the biological functions of EXOs for dealing with various diseases such as cancer, cardiovascular disorders, and neurological syndromes. However, the used dosages of EXOs are inconsistent, which vary with differences in experimental animal species, delivery methods, and kinds of diseases [42]. Several parameters were established and employed for dosing EXOs. For instance, total protein levels, total lipid levels, global RNA contents, and particle numbers are all used for quantifying amount of EXOs [42]. By considering the possibility of contamination of protein and lipids during exosome preparation, particle numbers are widely used for dosing EXOs [42]. In the present study, we also used particle numbers for calculating the dosage of EXOs for treating cartilage defects in rabbits. To select an appropriate dosage, we first examined the effects of EXOs at different dosages on cell viability, proliferation, and migration. Our data showed that 1 × 10^9^ particles/ml is a suitable dosage in cultured primary chondrocytes. Due to reduced bioavailability *in vivo*, a higher dose (1 × 10^10^ particles/ml or 5 × 10^10^ particles/ml; 30 *μ*l for each animal) was adopted for cartilage repair in rabbits, which was comparable to the dose of exosomes for treating osteoarthritis in mice [43]. Moreover, both studies used local administration of EXOs by intra-articular injection. To select an appropriate regimen, we analyzed the time course effects on exosome internalization in rabbit primary chondrocytes. We found that exosome internalization starts at 3 h incubation, and it gradually increases along with the time elongation and peaks at 72 h. Due to severe overlap of cells, we did not observe exosome internalization for longer time. Based upon these data, we conclude that the internalization of hBMSC-EXOs in chondrocytes may peak at 3-4 days after treatment, indicating hBMSC-EXOs could last for 6-8 days. Therefore, we treated rabbits with prepared EXOs once a week for 4 weeks. With this regimen, the prepared hBMSC-EXOs were directly injected into the articular cavity. Functional assays showed that osteochondral defects were largely repaired by hBMSC-EXOs. In line with our findings, several reports also have shown that EXOs from different MSCs have benefits in cartilage repair [20–23, 35].

In general, EXOs act as cargo for delivering various substances such as nucleic acids, proteins, and lipids to recipient cells and thus play their functions [44]. For example, Zhang et al. found that MSC-derived exosomal CD73 stimulates AKT and ERK signaling to increase cell proliferation and infiltration in chondrocytes during cartilage repair [35]. In addition to exosomal proteins, exosomal nucleic acids including miRNAs and long noncoding RNAs (lncRNAs) were extensively examined in cartilage regeneration. Wu et al. showed that miR-100-5p was enriched in MSC-EXOs, which inhibits mTOR signaling and thus attenuates articular injury in osteoarthritis [43]. lncRNA KLF3-AS1 was highly expressed in MSC-EXOs, and it suppresses IL-1*β*-induced apoptosis in chondrocytes [23, 32]. Based upon these findings, we proposed that hBMSC-EXO-mediated cartilage repair in the present study is likely due to some specific proteins, miRNAs, and/or lncRNAs in EXOs. Nevertheless, lipids and some other metabolites present in hBMSC-EXOs may also play a role in chondrocyte proliferation and extracellular matrix synthesis in cartilage repair. One project aimed at this topic is ongoing, in which combined technologies including RNA-seq, lipidomics, and proteomics will be employed to explore the underlying mechanisms.

In conclusion, in the present study, we prepared exosomes from hBMSCs to treat primary chondrocytes *in vitro* and rabbits with cartilage defects *in vivo*. Our data showed that hBMSC-EXOs improve cell viability, proliferation, and migration in primary chondrocytes. Meanwhile, hBMSC-EXOs also reduce cell apoptosis *in vitro*. In rabbits with cartilage defects, the application of hBMSC-EXOs largely promotes cartilage repair. These data strongly suggest that hBMSC-EXOs hold great therapeutic potentials for treating cartilage dysfunction-associated diseases. Moreover, these benefits are likely due to improved cellular functions in chondrocytes induced by hBMSC-EXOs.

However, the present study still includes several limitations. First, the observed benefits of hBMSC-EXOs in cartilage repair remain to be validated in more experiments using other animal models. Second, the mechanisms responsible for hBMSC-EXO-induced cartilage repair are still not clear, although we observed hBMSC-EXOs improve cell proliferation and migration in chondrocytes. The involved mechanisms will be elucidated by analyzing the constituents in prepared EXOs and related functional studies.

## 5. Conclusions

Overall, in the present study, we prepared exosomes from human bone marrow MSCs, which were then used to treat rabbits with osteochondral defects. Our data showed that these prepared exosomes greatly improved cartilage repair after injury. These benefits are likely due to increased cell viability, proliferation, mitochondrial function, and cell migration in chondrocytes induced by exosomes. All these data strongly suggest that exosomes derived from bone marrow MSCs hold great therapeutic potentials for treating cartilage dysfunction-associated diseases such as osteoarthritis and traumatic joint injury.

## Figures and Tables

**Figure 1:** Characterization of human bone marrow stromal cell- (hBMSC-) derived exosomes (EXOs). (a) Representative transmission electron microscope (TEM) images of hBMSC-EXOs (scale bar = 200 nm). (b) Nanoparticle tracking analysis for hBMSC-EXOs. (c) Western blots showing the exosome markers including CD81, TSG101, and Flotillin 1. *β*-Actin was used as a negative control. (d) Identification of rabbit chondrocytes. Cell morphology was observed at bright field with a microscope (scale bar = 100 *μ*m). Collagen II (COL II; red) was analyzed by immunofluorescence. DAPI (blue) was used to designate the nuclei. Scale bar = 50 *μ*m. (e) Internalization of hBMSC-EXOs in primary rabbit chondrocytes. hBMSC-EXOs were labeled by PKH26 (red) and incubated with primary chondrocytes. FITC-Phalloidin (green) and DAPI (blue) were used to label the cytoskeleton and the nucleus, respectively. Scale bar = 25 *μ*m.

**Figure 2:** hBMSC-EXOs improve cell viability and proliferation in chondrocytes. Rabbit primary chondrocytes were treated with hBMSC-EXOs at different dosages as indicated. 24 h or 48 h posttreatment, cell proliferation and cell viability were examined. (a) Cell viability was increased by hBMSC-EXOs in chondrocytes. CCK-8 assay was used to analyze cell viability. *n* = 3. (b) Cell proliferation was enhanced by hBMSC-EXOs in chondrocytes. Cell proliferation was assayed by EdU incorporation. *n* = 3. Scale bar = 400 *μ*m. (c) Quantitative analysis for EdU incorporation as shown in (b). Values are presented as mean ± SEM. ns means no significance. ^∗^*P* < 0.05 and ^∗∗∗^*P* < 0.001, versus the control group, one-way ANOVA.

**Figure 3:** hBMSC-EXOs promote cell migration and mitochondrial function in chondrocytes. Rabbit primary chondrocytes were treated with hBMSC-EXOs at 1.0 × 10^9^/ml for 24 h or 48 h. Cell migration and mitochondrial membrane potential were assayed. (a) hBMSC-EXOs stimulate cell migration. Wound healing assay was used to evaluate cell migration. Scale bar = 100 *μ*m. (b) Quantitative data for wound healing assay as shown in (a). (c) hBMSC-EXOs increase the mitochondrial membrane potential. Representative fluorescence images for JC-1 staining were shown. Scale bar = 100 *μ*m. (d) Quantitative analysis for JC-1 staining as shown in (c). *n* = 3. Values are presented as mean ± SEM. ^∗^*P* < 0.05, ^∗∗^*P* < 0.01, and ^∗∗∗^*P* < 0.001, versus the control group, one-way ANOVA.

**Figure 4:** The time course effect of hBMSC-EXO internalization in chondrocytes. (a) EXO internalization was gradually increased along with the time elongation. hBMSC-EXOs were labeled with PKH26 (red) and incubated with primary rabbit chondrocytes at the dosage of 1 × 10^9^/ml. Immunofluorescence staining was performed at different time points as indicated. FITC-Phalloidin (green) and DAPI (blue) were used to label the cytoskeleton and the nucleus, respectively. Scale bar = 50 *μ*m. (b) The fluorescence intensity for PKH26. *n* = 3. Values are presented as mean ± SEM. ^∗∗∗^*P* < 0.001, versus the control group, one-way ANOVA.

**Figure 5:** hBMSC-EXOs promote cartilage formation after injury in rabbits. (a) The experimental design. Defects were generated in the articular cartilage of rabbits, and then, hBMSC-EXOs were given to rabbits via intra-articular injection for 4 times. (b) The gross appearance of rabbit articular cartilages. (c) H&E staining. Scale bar = 1000 *μ*m. EXOs-low: 1 × 10^10^/ml; EXOs-high: 5 × 10^10^/ml.

**Figure 6:** hBMSC-EXOs promote cartilage repair in rabbits. (a) Saf-O/Fast Green staining. Scale bar = 1000 *μ*m. (b) The International Cartilage Repair Society (ICRS) scores. *n* = 3. Values are presented as mean ± SEM. ^∗^*P* < 0.05, ^∗∗^*P* < 0.01, and ^∗∗∗^*P* < 0.001, one-way ANOVA. EXOs-low: 1 × 10^10^/ml; EXOs-high: 5 × 10^10^/ml.

## Data Availability

The data that support the findings of this study are available from the corresponding author upon reasonable request.
